# Efficacy and Adverse Reactions of Arthroscopic Half-Moon Plate Invasive Surgery in Patients with Acute Knee Pain (AKP): Systematic Review and Meta-Analysis

This article has been retracted.

**DOI:** 10.1155/2022/4277563

**Published:** 2022-04-18

**Authors:** Luping Sun, Zhidan Huang

**Affiliations:** ^1^The Fifth Central Hospital of Tianjin, China; ^2^The People's Hospital of Puning, Pharmaceutical University, China

## Abstract

**Objective:**

To evaluate the efficacy and adverse reactions of arthroscopic half-moon plate invasive surgery (DEB) in patients with knee pain (AKP) using meta-analysis techniques.

**Methods:**

The computer retrieves from the English databases PubMed, EMBASE, Cochrane Library, and Web of Science and the Chinese databases China Knowledge Network, Wanfang Database, VIP Database, and China Biomedical Literature Database to collect information about DEB therapeutic AKP randomized controlled trial. Develop criteria for documentation inclusion and exclusion, evaluate the quality and bias risk of literature, and compare differences in efficacy and adverse responses before and after DEB treatment and other conservative treatments.

**Results:**

A total of 14 randomized controlled trials and 1464 AKP patients were included in the study, with follow-up duration of 1-12 months. The total knee scores for DEB at 1, 3, 6, and 12 months after treatment were significantly better than baseline levels (1 month: WMD = 34.56, *P* = 0.02; 3 months: WMD = 27.73, *P* = 0.0001; 6 months: SMD = 2.38, *P* = 0.0001; 12 months: SMD = 1.69, *P* = 0.001). At 6 months of follow-up, DEB improved knee function better than HA (SMD = 0.47, *P* = 0.003), and during follow-up for 12 months, DEB relieved knee pain (SMD = 0.55, *P* = 0.0007) and improved knee function (SMD = 0.88, *P* = 0.0001) which is significantly better than HA. DEB was less effective at improving knee function in 1, 3, and 12 months than DEB joint HA injections (1 month *P* = 004; 3 months *P* = 0.01; 12 months *P* = 0.03). At 6 and 12 months of follow-up, DEB was better at pain relief and improved function than ozone (*P* > 0.05). DEB and glucocorticosteroids have similar effects in pain relief and improved function at various follow-up times. In terms of adverse reactions, DEB does not increase the risk of adverse events compared to HA (OR = 0.96, *P* = 0.85).

**Conclusion:**

Compared to HA and ozone, DEB is a more effective treatment for AKP joints, while DEB is combined with HA. The clinical efficacy of injection therapy AKP is better than that of DEB alone.

## 1. Introduction

Knee pain (acute knee pain (AKP)) is a chronic degenerative disease caused by factors such as chronic degeneration of the knee joint, trauma, and overwork of the knee joint. The main pathological features of the disease are joint cartilage damage, reactive hyperplantation of the lower bone of secondary cartilage, and inflammation of the sliding membrane and can affect the entire joint and the tissue around the joint. Because of the complex pathological mechanism of AKP, high incidence and high disability rate, it will bring huge medical economic burden to the whole society, so it has become a hot topic in clinical research.

Pain is a self-protection mechanism of the human body; with the gradual progress of society and the further extension of human life, chronic pain caused by medical and social problems is gaining more and more attention; there are experimental results showing that the nerve fibers responsible for transmitting damaging information exist in the incoming nerve fibers; more sensitive to mechanical stimulation A6 nerve fibers are responsible for conducting rapid pain. The main chemical stimulation can also include mechanical and temperature stimulation which is more sensitive to the class C nerve fibers mainly responsible for the transmission of slow pain; studies show that deep tissue, including bone membranes, joint sacs, ligaments, muscles, and other deep tissue, have mainly slow pain [1].

The neural domination of joints is described in relative detail; they think that joint sacs, ligaments around joints, and their attachment points are relatively rich in nerve control, but also more nerve fibers distributed close to the joint edge of the bone membrane, knee slip membrane, and cartilage lower bone blood vessels. Wyke considers as a nonspherical IV nerve ending; C fiber is responsible for knee pain, it is present as interstitial and plexus around blood vessels and free nerve endings form located in the knee joint sac, sliding membrane, and joint fat pad, but the above-mentioned receptors are not active under normal circumstances, only when joint tension significantly increased or stimulated by chemicals; these chemicals are roughly lactic acid, neuropeptides, histamines, excitation, and prostatin. Therefore, most scholars believe that knee pain is caused by a joint effect of chemical and mechanical stimuli. Joint cartilage is not neural distribution, so the injury will not directly produce pain, but cartilage under the bone, bone membrane, sliding membrane, ligament, and joint sacs have a rich neural distribution, which also constitutes the source of pain stimulation of knee-off osteoarthritis [2].

An important feature of knee osteoarthritis is glial gliosis, and inflammation of the membrane can lead to pain in knee osteoarthritis, known as “inflammatory pain.” It has been suggested that secondary gliosis may be caused by bone fragments and other “joint debris.” Calcium-containing crystals, including alkaline calcium phosphate and calcium dihydrate pyrophosphate, can lead to the development of gliosis, while the accumulation of neuropeptides can further aggravate inflammation of the membrane. Primary damage to the joint sensory neurons in the cell can synthesize and release chemicals that regulate the chemical environment of their peripheral ends, which are transported through axial slurry to the end of the peripheral nerve and released in the event of depolarization. Damaged cells and tissues at the site of the injury release chemicals such as P substances, histamines, prostaglandins, and white triene to make peripheral injury receptors sensitive, which can reduce the threshold of excitement of the injury receptor or activate the injury receptor directly. Neurogenic inflammation acts on slip membranes, blood vessels in joint sacs, fat cells, mononucleosis-macrophages, fibroblasts, and membrane cells (which have SP receptors on these cells). Neuropeptides such as P-substances of a G protein and calcitonin-based anticalcitonin, which act on blood vessels, etc., are called “neurogenic inflammation” due to related peptides [3].

The nerves that make up the knee joint can be divided into shallow and deep layers; the frontal cortex nerve and the femal epithelial nerve are the shallow layers of the nerves that make up the knee joint. The joint branch is deep. As shallow cortex nerves, the femal cortex nerve, the femal epithelial nerve, the closed-hole nerve, and the hidden nerve are interspersed in the front, rear, and inner part of the knee. We can generally distribute the ligaments around the joint, the joint sac, and the intrajoint into the joint into four groups: the first group is the nerve endings that govern the quadriceps, and the joint sacs distributed near the upper edge of the tibia are called the upper region group of the bones The ligaments of the lower part of the lower part of the shin and the front and knee joints, the joint sacs, and the subcutaneous fat pads and the pre-cross-ligaments that dominate the joints, respectively, are distributed by the hidden nerve branches, known as the inner and lower ligament groups. The nerves distributed in the outer fat pads and joint sacs are composed of the exostretchal ligament nerve and the phosphate, Phoebe deep nerve joint back stretched Phoebe's total nerve branch, which is called the outer region group nerves, sciatic nerves, closed-hole nerve branches form a group called argon region and cross them into the joints to dominate the post-cross-ligaments; the above four groups of nerve distribution overlap but the dominant area has a clear division and formation of most of the body nerves in the joint and its autonomic neural network [4].

For severe AKPs, knee replacement surgery is an effective solution, with more conservative treatment options for mild and moderate AKP patients. However, there are currently very limited clinical conservative treatments for AKP, mainly nonsteroidal anti-inflammatory drugs (NSAIDs) and intrajoint injections of hyaluronic acid (HA), ozone, and hormone drugs. Although these drugs can improve patient function and reduce pain in the short term, there is no evidence that these drugs can improve the AKP process [5].

This study, through a comprehensive search of the relevant randomized controlled trials of DEB treatment AKP, used systematic evaluation and meta-analysis to reveal the effects of injection of other drugs before and after DEB treatment and in the DEB and joint cavity differences in pain relief and improved joint function in AKP patients, as well as in comparing the differences in adverse reactions of various joint injection drugs, providing a basis for clinicians to more standardized and reasonable application of DEB to treat AKP [6].

## 2. Methods in Treating AKP

The conventional treatment of knee osteoarthritis can be broadly divided into physiotherapy, drug therapy, intrajoint injection therapy, surgical treatment, and other related treatment methods; physiotherapy also generally includes epithelial nerve point stimulation therapy, electromagnetic field therapy, ultrasound therapy, low-dose laser therapy, cartilage radiofrequency forming, bivinegar Rein, calcitonin, sulfate amino glucose and chondroitin sulfate, dimethyl phosphate, diphosphate and traditional Chinese medicine treatment internal injection therapy, radiation colloidal intracanal injection therapy, surgical treatment routine including arthroscopic knee cleansing, autologous cartilage transplantation, autologous cartilage cell transplantation, artificial half-moon board replacement surgery, tibia high bone amputation, and section replacement. Other treatments include cytokine therapy, gene therapy, metal protein inhibitors, nitric oxide, and weight loss. Upon the appearance of knee osteoarthritis, first choose the appropriate rest, weight loss, limp and drug treatment, and other conservative therapy; when the symptoms are gradually serious enough to be in remission and after conservative treatment without obvious effect, at this time, patients usually consider the choice of surgical treatment; in the past, patients' standing advice is knee incision and force line correction surgery at the near end of the tibia or the far end of the femur, but at this time, the patient's knee pathological changes are often very serious; if arthritis further worsens, the patient will eventually be difficult to avoid artificial joint replacement. But most patients are reluctant to undergo surgery that is more damaging. Until the emergence of arthroscopic surgery, the treatment of osteoarthritis has achieved a breakthrough [7].

### 2.1. Arthroscopic Surgery Treatment

Studies have shown that at any stage of knee osteoarthritis is suitable for closed-sectional surgery; arthroscopic surgery compared with the previous use of surgery, the treatment costs are lower, trauma is small, recovery is fast, it is repeatable, there are fewer complications and other advantages, and patients have reduced or even avoid long-term use of nonsteroidal anti-inflammatory analgesic drugs, which can reduce damage to the gastrointestinal tract and other side effects.

### 2.2. Joint Cleansing

During surgery, by cleaning up cumbersome bone that may cause pain affects the normal movement of the knee joint and may wear out the normal structure of the knee joint; trim or remove the half-moon plate, flatten the joint surface, remove the free body, and release preoperative examination and observation during surgery to find the outer support band with contractions [8].

### 2.3. Free Body, Removal of Hyperplastic Bone, and Trimming of Cartilage

Bone formed by proliferation between femurs may narrow the interdental nest and in the activity of the knee joint with the tibia. The impact of bone hyperplasia of interstitial ratchet causes knee-tight mobility disorder; we can find that such patients are often clinically manifested as knee flexor malformation, further leading to patients and standing position when the knee joint cannot be fully straightened and presented as arch bridge-like changes; in this case, there are less scholars to study it and found that femur interstitial enlargement molding to remove bone can be different degrees of correction of the internal and external deformities of the joint, making it an effective method in the treatment of knee osteoarthritis and through cartilage dressing can promote the repair of cartilage and prevent gradual freeing and formation of intrajoint free body. In the late stages of degenerative arthritis can also be seen the formation of free bodies of varying sizes; most of these free bodies are considered by mathematicians to be cartilage source, that is, cartilage fragments peeling may also be bone cartilage source, from the peripheral bone or along the membrane; these free pieces usually occur between the joint surface and cause pain; this study through free body, the removal of proliferating bone custrum, and cartilage dressing can effectively reduce the device-derived pain and also can improve function [9].

### 2.4. Dressing of the Half-Moon Plate

Clinically found in the elderly patients and patients with advanced arthritis to degenerative tearing of the half-moon plate, while the majority of young people to traumatic tearing, at this time some scholars advocate the use of minimally invasive methods for the treatment of the degenerative half-moon plate. Clinically, it has been found that, for knee osteoarthritis, semimoon plate degeneration tearing and low quality of life requirements of patients with arthroscopic arthritis as a better palliative treatment method, but this method is not suitable for use under certain circumstances that has certain limitations, especially for patients with advanced knee osteoarthritis and the presence of knee joint malformation or severely narrow joint clearance. Repairing the half-moon plate further reduces its irritation to the slip film and the damage part of the card pressure that appears in joint movement [10].

### 2.5. External Support with Loosening

The femur joint as an important component of the knee joint in most patients with knee-off osteoarthritis has different degrees of injury performance; in the pathogenesis, it can be considered to be the cause of various factors leading to abnormal anatomy and mechanics of the femur joint can cause abnormal contact so that the local stress of the femur joint surface increases or decreases so that the pressure distribution is uneven, further leading to joint cartilage damage. In the reports related to knee osteoarthritis and arthritis arthroscopic treatment, there are many ways to solve the abnormality of the anatomical and mechanic characteristics of the femur joint: the comprehensive treatment method such as biting off femur hyperplasia, cutting pathological changes of the joint surface, and loosening the outer support belt has significant effect on the treatment of femur arthritis. It is reported that the loose outer support band under arthroscopic has obvious effect on knee pain and joint dysfunction caused by arthritis, with an excellent rate of up to 77%. This study can effectively improve the anatomical and mechanic characteristics of the femur joint abnormalities [11].

### 2.6. Joint Cleansing

Both groups in this study performed continuous flushing of the joint cavity simultaneously through arthroscopic surgery to remove inflammatory media and inflammatory proteins, reduce pressure in the knee cavity, and regulate and improve the knee cavity acidity and the role of osmotic pressure, clinically found that the knee's inflammatory slip membrane through the arthroscopic removal can directly reduce the knee-slip membrane inflammation on the knee erosion effect, but it also can remove inflammatory factors and reduce cytokines into the blood circulation, thus reducing the damage caused to other joints; this study of sliding membrane removal can effectively reduce the above-mentioned “inflammatory pain,” but it is also an effective prevention of knee erosion [12].

### 2.7. The Theoretical Basis for Denaturation

To improve knee arthritis dysfunction and pain, some scholars believe that the pain from the nerve sources of the knee is mainly the front, side, and rear of the femur; the research team through the mirror electric knife burned the nerves around the tibia to deneurize. The lower end of the femur, including the front, side, and rear of the femur and the electrocution of the joint sac attachment, is de-deenergized and deneuroticized 5-10 cm, effective in reducing the number of harmful sensory neurons and the neuropeptide substances released by them, thereby reducing the factors associated with pain, and because the tibia nerves overlap with each other and are composed of different components, so even if cut off, will not completely block the nerve support of the tibia nerve to the tibia, which will not seriously affect the permanent loss of skin sensation around the tibia; there are studies which show that the tibia cartilage around the electric cut plexus does not damage the preskull tissue. The vascular holes in the tibia are mainly located in the upper and lower quarter of the area of the tibia, so they do not cause complications such as tibia fractures and necrosis [13].

## 3. Materials and Methods

### 3.1. Document Retrieval Strategy

Computers retrieve from English databases PubMed, EMBASE, Cochrane Library, and Web of Science and Chinese databases China Knowledge Network (CNKI), Wanfang, VIP Database, and the Chinese Biomedical Literature Database (CBM). Retrieval is a combination of subject and free words, which is retrieved by connecting Boolean logic operators. Search terms include “Osteoarthritis”, “Osteoarthritides”, “Osteoarthroses”, “Arthritis, Degenerative”, “Arthritides, Degenerative”, “Degenerative Arthritides”, “Degenerative arthritis”, “Osteoarthrosis Deformans”, “Platelet-rich plasma”, “Plasma”, “Platelet-Rich”, “Platelet Rich Plasma”, “DEB”, “Randomized controlled trials”, “Osteoarthritis”, “Degenerative arthritis”, “Degenerative arthritis”, “Osteoarthritis”, “Platelet-rich plasma”, “DEB”, “Platelet”, “Plasma”, “Growth factor”, “Random”. The search deadline is September 2018 and manually searches documents that may meet the inclusion criteria by reading the literature [14].

### 3.2. Criteria for the Inclusion and Exclusion of Literature

The literature includes criteria (1) study type: randomized controlled trial; (2) subject: diagnosed with knee osteoarthritis patients; (3) dry premeasures: the experimental group (DEB) and control group have intracavocal injections.

Literature exclusion criteria: (1) nonrandomized controlled trials; (2) DEB combined oral medicine, traditional Chinese medicine, or surgical treatment; (3) incomplete literature data or contact with the author cannot be extracted; (4) repeated publication of the literature.

### 3.3. Literature Screening, Extract Analysis, and Bias Risk Assessment

The titles and abstracts of the literature, which were published by 2 researchers reading the retrieval strategy, were independently extracted according to preset criteria for inclusion and exclusion. It was eventually determined by three researchers that the final inclusion was made in the literature [15]. The extract was conducted independently by two researchers, who were divided and the 3rd researcher was involved in the discussion. The extraction of literature includes (1) literature title, first author, and year of publication and (2) sample size, follow-up time, main observation indicators, and adverse reactions in each group of subjects. For literature that takes different or multiple knee function scores, it is according to the Osteoarthritis Index of the University of Xi'an and McMaster.

Western Ontario and McMaster Universities Osteoarthritis Index (WOMAC) knee injury and osteoarthritis rating criteria (knee injury and osteoarthritis outcome score (KOOS)) and International Knee Documentation Committee Score (IKDC) prioritize the extraction of data. For literature that adopts the same scoring criteria, the weighted mean deviation (WMD) is calculated as a summary analysis of the effect amount, and for literature that describes the same result by different scoring criteria, the standardized mean difference is calculated (SMD) providing a summary analysis of the amount of effect, and after a summary analysis of adverse reactions in each study, the relative risk (RR) is calculated [16].

### 3.4. Bias Risk Assessment

The assessment was independently conducted by 2 researchers based on Cochrane bias risk assessment criteria, including (1) random number generation (selective bias), (2) allocation result hiding, (3) patient blindness (implementation bias), (4) result evaluator blindness (measurement bias), (5) incomplete result data (missed access bias), (6) selective result reporting (report bias), and (7) other bias.

Each item in the literature is low-risk bias, which is considered to be low-risk bias. Items 1-2 are high-risk bias or uncertainty, moderate bias, and more items are high-risk bias or uncertainty and are considered highly biased.

### 3.5. Statistical Analysis

Meta-analysis is performed using RevMan 5.3 software and Stata 14.0 software from the Cochrane Collaboration Network. The heterogeneous size is determined by the statistical value *I*^2^ for quantitative analysis; when *I*^2^ is 25%, 50%, and 75%, it represents low, medium, and high heterogeneity, respectively. When *I*^2^ < 50%, a fixed-effect model is used, and when *I*^2^ > 50%, analyzing heterogeneous sources, the random-effect model is used. We use Egger tests to evaluate publication bias. When the *P* value < 0.05, the result is considered statistically significant [17].

### 3.6. General Situation Included in the Study

We obtained a total of 707 documents through Chinese and English database retrieval and manual search. Three researchers screened, first and rescreened, and the final 14 literatures were identified for inclusion in the study for quantitative analysis.

The documentation is included in the process. In the 14 randomized controlled trials included, a total of 1464 AKP patients were included in the study's control group and the patients' gender, age, and weight. There was no significant difference in course of disease and clinical symptoms. 14 studies were included, 10 compared the efficacy of DEB with HA in AKP patients. The study compared the efficacy of DEB with DEB combined HA, and two studies compared the efficacy of DEB with glucocorticosteroids; 1 study compared the clinical effects of DEB with ozone. In terms of the severity of the classification of AKP, a total of 12 studies used the Kellgren-Lawrence scale, and 1 study used Ahlback scales; in addition, 1 study was not reported [18].

### 3.7. Bias Risk Assessment Incorporated into the Literature

Our literature risk bias assessment based on the Cochrane bias risk assessment criteria showed that there were 9 moderate bias literatures and 5 highly biased literatures. We used the Egger test to detect publishing bias, and the results showed no evidence of significant publishing bias.

## 4. Results

### 4.1. Comparison of Efficacy before and after DEB Treatment of AKP

In 1 month after DEB treatment, 2 studies compared the total knee score of AKP patients with baseline changes, and the combined result analysis showed that the total knee score of patients improved significantly compared to pretreatment: (WMD = 34.56; 95% CI 5.07, 64.06; *P* = 0.02); the result is significantly heterogeneous (*I*^2^ = 99%) (Figure 1). In the 3 months after DEB treatment, three studies compared the total knee score of AKP patients with baseline changes, and the results showed that the total knee score of patients improved significantly compared to pretreatment (WMD = 27.73; 95% CI 14.15, 41.31; *P* = 0.0001); the results are significantly heterogeneous (Figure 2). Six months after DEB treatment, 10 studies compared the total knee score of AKP patients with baseline changes, and the results showed that the total knee score of patients was significantly improved compared to pretreatment levels (SMD = 2.38; 95% CI 1.18, 3.58; *P* = 0.0001); the result has a significant heterogeneity (*I*^2^ = 98%). In 12 months after DEB treatment, 8 studies compared the total knee score of AKP patients with baseline changes, and the combined results showed that the total knee score of patients also improved significantly compared to before treatment (SMD = 1.69; 95% CI 0.69, 2.69; *P* = 0.001). The results are significantly heterogeneous (*I*^2^ = 97%) (Figure 3). The increase in score was most pronounced in 1 month after DEB treatment and decreased gradually with the extended treatment time, but the difference in baseline level was statistically significant [18].

In terms of knee pain scores, 8 studies used WOMAC pain scores and two used KOOS pain scores. A total of five studies compared the efficacy of DEB and HA in relieving knee pain 1 month after treatment, and the combined results showed that HA was superior to DEB in relieving knee pain, but the difference was not statistically significant (SMD = 0.31; 95% CI -0.12, 0.73; *P* = 0.16); the result is significantly heterogeneous (*I*^2^ = 73%) (Figure 4). A total of four studies compared the efficacy of DEB and HA in relieving knee pain in three months after treatment, and the combined results showed that HA was better than DEB in relieving knee pain. However, the difference is not statistically significant (SMD = 0.17; 95% CI -0.34, 0.67; *P* = 0.52); the result is significantly heterogeneous (*I*^2^ = 68%) (Figure 5). A total of eight studies compared the effects of DEB and HA on improved pain over the last six months of treatment, and the results showed that DEB was superior to HA in improving knee pain in patients. However, the difference is still not statistically significant (SMD = 0.34; 95% CI -0.69, 0.01) [19].

### 4.2. DEB Compared to HA's Efficacy and Adverse Reactions

In terms of knee pain scores, there were eight studies using WOMAC pain scores and two USKOS pain scores. A total of five studies compared the efficacy of DEB and HA in relieving knee pain 1 month after treatment, and the combined result analysis showed that HA is better than DEB in relieving knee pain, but less statistically significant (SMD = 0.31; 95% CI -0.12, 0.73); the result is significantly heterogeneous (*I*^2^ = 73%). A total of 4 studies compared the efficacy of DEB and HA in relieving knee pain 3 months after treatment, and the combined result analysis showed that HA is superior to DEB in relieving knee pain, but the difference is not statistically significant (SMD = 0.17; 95% CI -0.34, 0.67; *P* = 0.52); the fruit is significantly heterogeneous (*I*^2^ = 68%) (Figure 6). A total of eight studies compared the effects of DEB and HA treatment on improved pain over the next six months, and the results showed that DEB is superior to HA in improving knee pain in patients, but the differences are still not statistically significant (SMD = 0.34; 95% CI -0.69, 0.01; *P* = 0.06); the result is significantly heterogeneous (*I*^2^ = 82%); a total of 8 studies compared DEB with HA after treatment [20] (Figure 7).

## 5. Discussion

Traditional arthroscopic knee cleansing to treat knee osteoarthritis has a certain effect. Arthroscopic knee cleansing combined with denaturation to treat knee osteoarthritis can significantly improve the effectiveness of treatment. One year after surgery than the traditional arthroscopic knee cleanup rate has significantly improved [21]. The combined denaturation long-term efficacy of traditional arthroscopic knee cleansing and arthroscopic knee cleanup is to be further studied after long follow-up [22].

This study reduced the factors affecting the efficacy of arthroscopic surgery. In addition to surgical techniques and postoperative rehabilitation training, there are other factors, such as age, surgery time, psychological factors, postoperative rehabilitation training, the application of hemorrhage belt, and postoperative joint hematopoietic buildup. There is literature that is less than 65 years old, the disease history is less than 10 years of good results, there is also literature that studies arthroscopic surgery effect and age is not relevant, the above two studies are still academically controversial, but it is certain that older patients should try to avoid surgical treatment if there is no special necessity; otherwise, it may cause additional pain to patients, so this study included age. Patients aged 35~65 were the subjects of studies that showed an inverse relationship between the length of surgery and the efficacy of surgery and that surgery that took too long or more than 90 minutes under arthroscopic treatment was not ideal. We believe that this is due to extensive joint cleansing and prolonged intrajoint operation which can not only aggravate damage in the joint and increase fluid seepage and bleeding in the joint sac. Joint cleansing is not the ultimate treatment, which cannot fundamentally solve the reduction of knee pain and improve the function of the knee joint, so this kind of surgery needs to reduce the trauma to the lowest possible level, so we should be fully prepared before surgery, so as to minimize the time of surgery; of course, it depends more on the proficiency of the lead physician, because this study included less than 90 minutes of surgery time. Some patients have high expectations for arthroscopic surgery, often leading to dissatisfaction with the postoperative efficacy, so patients and their families should be detailed before surgery. Knowing the nature and expected effect of the procedure, in accordance with the principle of individual treatment according to the specific situation, and abiding by the principle of gradual progression, after surgery, the patient should be guided to carry out early knee activity to promote blood circulation and lymphatic reflux, thereby reducing tissue edema, which is conducive to the recovery of tissue metabolism and joint function activities.

The application of hemostatic band should strictly abide by the use of norms; although there are reports that the use of the hemorrhage band is too long, there are cases of surgical paralysis, and there are often reports that the use of hemorrhage band will aggravate the swelling of the surgical limb, but the application of hemostatic band can effectively reduce blood during surgery; all surgical patients in this study have applied hemorrhage band hemorrhage to ensure clear surgical vision. In order to reduce postoperative joint swelling, limited movement, etc. caused by postoperative joint hemorrhage, the subjects of this study applied radiofrequency instrument to intrajoint hemorrhage, and after surgery, elastic bandage pressure bandages and other effective methods were used to reduce intrajoint blood accumulation [23–25].

The limitations of this technique include an inability to own long follow-up time, as arthroscopic knee cleanup joint deneuroticization was carried out. The long-term efficacy has yet to be further studied. Whether the procedure can replace knee replacement or significantly less replacement rate is subject to long-term follow-up and further study.

Overall, we rated the strength of evidence for efficacy of auriculotherapy compared to control for the treatment of pain as moderate. This was based on the magnitude of the mean differences we found overall and for each subgroup, the high consistency in direction and magnitude of effects noted throughout the studies, the lack of evidence of publication bias, the preponderance of good and fair quality studies, and the stability of our estimates with poor quality studies removed. Although we acknowledge the generally low strength of evidence of efficacy for acute and chronic pain subcategories, we note that the direction of effect appears to favor efficacy of auriculotherapy.

## 6. Conclusion

Compared to HA and ozone, DEB is a more effective treatment for AKP joints, while DEB is combined with HA. The clinical efficacy of injection therapy AKP is better than that of DEB alone, which may be further applied in the clinic in the future.

## Figures and Tables

**Figure 1:** PRISMA study over the study methods.

**Figure 2:** Comparing the total knee score of AKP patients with baseline changes.

**Figure 3:** AKP patients with baseline changes of 2 months after DEB treatment.

**Figure 4:** DEB compared to HA's efficacy and adverse reactions.

**Figure 5:** Comparing the efficacy of DEB and HA in relieving knee pain three months after treatment.

**Figure 6:** Comparing the efficacy of DEB and HA in relieving knee pain 3 months after treatment.

**Figure 7:** An overview of the methodological quality results. Risk of bias and applicability concern graph.

## Data Availability

The data used to support this study is available from the corresponding author upon request.
